The article "Problems and Countermeasures of College Students' Mental Health Education" was published in 2022. Journal: J Healthc Eng.

# Problems and Countermeasures of College Students' Mental Health Education

**DOI:** 10.1155/2022/6430855

**Published:** 2022-01-11

**Authors:** Xiaoli Zhang

**Affiliations:** Guangdong Institute of Petroleum and Chemical Engineering, Maoming, Guangdong 525000, China

## Abstract

Compared with the previous teaching environment and model, college students need more self-awareness and self-discipline to learn better. In order to solve many mental health problems of college students, this work studies that the school should increase policy support to relevant parties and strengthen the cultivation of college students' psychological counseling ability, so as to provide more psychological counseling services for college students. This work studies and analyzes the common problems in contemporary college students' mental health education, such as lack of teachers, mere formality, imperfect system, and poor pertinence, and puts forward the corresponding countermeasures for college students' mental health education. When college students enter the university, they need to further improve their knowledge and ability to achieve professional development in a relatively loose learning environment. University is a key period for college students' personality improvement and physical and mental development. With the increasing pressure of social employment, the psychological pressure of college students is increasing. This study provides a reference for the mental health problems of college students.

## 1. Introduction

Colleges and universities are the main positions to cultivate high-quality and comprehensive talents and also the main places for college students to live and study. In recent years, with the continuous expansion of college enrollment and the de elitism of higher education, higher requirements are put forward for college students' psychological quality and adaptability [1]. At present, with the fierce social competition and the increasingly severe employment situation, the mental health problems of college students are becoming more and more prominent [2]. At present, there are a series of problems in college students' mental health education, such as insufficient attention, lack of teachers, mere formality, single channel, imperfect system, and poor pertinence [3]. There is a general situation of self-closure among college students, and such college students occupy a considerable proportion in the national college students. As time goes by, some college students are not good at communicating with the outside world [4]. At present, a considerable number of students in colleges and universities have psychological problems and psychological confusion. Educators in colleges and universities gradually focus on the mental health education of college students, and the mental health rate of college students is also lower than that of ordinary college students at the same level [5]. College students' mental health education is not only related to their personal growth but also has a profound impact on the stability of colleges, families, and even the whole society.

Mental health is getting more and more attention in today's society, especially the problems of college students are constantly exposed. Mental health education has become one of the urgent problems in college education, and it is also the key content of college education [6]. In the relatively relaxed learning environment, college students need to further improve their knowledge and ability to achieve professional development. Compared with the previous teaching environment and mode, college students need more self-consciousness and self-discipline consciousness to learn better [7]. Although the mental health education in colleges and universities has achieved certain results, there are still some problems that cannot be ignored. We must take effective measures to find out the existing problems and actively explore new work ideas [8]. With the rapid development of society and the acceleration of the pace of life, the pressure of learning, emotion, and employment of contemporary college students is increasing, and the mental health education of college students cannot be ignored [9]. Under the pressure of the study, making friends, and job hunting, many college students have mental health problems. It has become an important topic for colleges and universities to explore and analyze college students' mental health problems and find solutions to them [10]. This study analyzes the common problems of mental health education of contemporary college students, such as lack of teachers, mere formality, imperfect system, and poor pertinence, and puts forward corresponding countermeasures for college students' mental health education.

## 2. The Problems of Mental Health Education for College Students

### 2.1. Poor Adaptability to Environment

Since the reform and opening up, with the integration of Chinese education with Western developed countries, college students' mental health education has paid more and more attention, but as far as the overall demand is concerned, this improvement is still far from enough. At present, the main forms of mental health education in colleges and universities include offering mental health education courses, conducting psychological consultation, conducting lectures on mental health education, and setting up psychological health education consultation rooms. Many of these forms cannot be carried out in depth due to the lack of attention and funds in colleges and universities, which makes these superficial forms unable to meet the basic requirements of mental health education for college students. Some colleges and universities lack correct understanding and research on the tasks, functions, characteristics, and laws of college students' mental health education under the new situation. At present, psychological counseling institutions established in colleges and universities have a variety of subordinate relationships, most of which are affiliated with student offices, while some are affiliated with youth league committees, propaganda departments, or school hospitals. College students are in a stage of interpersonal communication with rich self-development, but the current mental health education in colleges and universities lacks the cultivation of students' practical ability. Mental health education in colleges and universities is mainly implemented in the form of elective courses, lectures, and teachers' lectures. The teaching method is single and formal, lacking practicality and effectiveness. In the stage of university education, the content of mental health should be infiltrated into the teaching of various disciplines. However, there are not many requirements for the internal development of modern discipline teaching theory and practice. The teaching of various disciplines takes the cultivation and improvement of students' ability as the central task.

When college students encounter psychological problems in their life or study, they often confide to their relatives or friends around them and seldom think of seeking help from professional psychological counseling institutions in colleges and universities, so it is difficult to fundamentally solve the actual needs of the healthy development of college students' psychology. Compared with mathematics, Chinese, and other professional courses, the development history of mental health education courses is relatively late. In addition, the development of higher education in China is relatively late [11]. Although it has developed rapidly in recent years, it is still far behind the advanced countries, which leads to the lack of professionalism of educators. College students' mental health education teachers are weak. At present, the full-time mental health education teachers in colleges and universities are weak, which cannot meet the needs of the rapid development of higher education and the increasing psychological needs of students. The lack of professional mental health teachers is also a common problem in colleges and universities. As far as the reality is concerned, teachers in charge of students' mental health education are often served by counselors or teachers from other functional departments. Due to the lack of professional knowledge and multiple roles, the corresponding psychological guidance function cannot be well played, which is not conducive to the promotion of mental health education for college students.

### 2.2. Lack of Communication Skills

Mental health education course is one of the important ways to implement mental health education. At present, although there are many textbooks and books on mental health education for college students, most of them are not practical, and the versions are complicated. From the implementation of the curriculum, some colleges and universities regard mental health education as a course to impart psychological knowledge and teach students psychological concepts, principles, and other psychological knowledge too much, ignoring the cultivation of humanistic spirit and cultural accomplishment. Mental health education in colleges and universities is a scientific, normative, and operational work, which requires highly professionals, and only those who have undergone systematic and standardized training can be competent. On the whole, however, the professional level of mental health education teams in colleges and universities is uneven, and most teachers rush to work after short-term training, so they cannot track the students with psychological problems in time.

With the oversupply of college graduates, college students' realistic pressure and self-experience pressure are constantly increasing. As a result, many college students have more psychological confusion, and some people have anxiety, compulsion, and paranoia in their study and life. Mental health education and ideological and political education of college students are unified in terms of working objects, ultimate goals, and teaching methods, while they are essentially different in terms of their respective theories, methods, and operating mechanisms. College students' mental health education should be a systematic educational process. However, at present, most colleges and universities take students' mental health education as a part of ideological education, lacking a complete system [12]. Due to the limitations of mental health educators in learning network technology and loopholes in management, some college students' personal secrets and psychological privacy are not protected. Therefore, mental health education in colleges and universities should give full play to the role and advantages of network mental health education, promote the healthy growth of college students' psychology, make them meet the needs of society, and promote social harmony and stability.

## 3. Countermeasures for Optimizing the Mental Health Education of College Students

### 3.1. Improve the Incentive Mechanism

Colleges and universities should actively strengthen the construction of their own teachers, attract professional talents to settle in the university, and thus ensure the professionalization of teachers in mental health education. In this process, the education department, as a functional department, mainly focuses on policy guidance, and the concrete implementation depends on the conscious and active efforts of universities. Colleges and universities should organize experts as soon as possible to compile practical, operable, and interesting high-quality teaching materials in line with the psychological development of college students. The teaching of courses should take students' interests and psychological needs as the breakthrough point, combine with the characteristics of the times, and try to be close to students' reality to improve the attractiveness of mental health education. Environment plays an important role in people's psychological development, and a positive campus atmosphere can promote students' healthy growth. In view of this, colleges and universities should strengthen the construction of psychological education environment, increase investment in education, update the hardware and equipment of psychological education, do a good job in campus greening and beautification, and optimize the physical environment of campus, so that students can study and live in a clean, tidy, and comfortable environment [13]. While performing the duties of students' mental health education, colleges and universities should also set up mental health education consultation institutions, which are responsible for students' daily mental health education, consultation, and counseling, so as to help students clear their psychological barriers and solve their psychological confusion [14].

College students' mental health education is a systematic project. Colleges and universities should establish a sound organization, combine with other kinds of education, formulate relevant laws and regulations, and carry out college students' mental health education in the new period according to law. The formation of good psychological quality is not formed in a day, but needs long-term training. For example, Table 1 provides the investigation of psychological training plan.

Multichannel mental health education will undoubtedly serve more people to a certain extent and greatly improve the audience of psychological counseling. At the same time, we should analyze and summarize the various pressures faced by college students and conduct classified counseling in various forms. The interactive relationship of students' social development is shown in Figure 1.

The outbreak of college students' psychological crisis is characterized by suddenness and urgency, but it is difficult to accurately predict when it will break out and the degree of damage, which does not mean that it is unpredictable and helpless. Whether the external bad stimulus will cause psychological crisis depends on the inner psychological characteristics of college students.  Figure 2 shows the evolution structure of college students' psychological crisis.

Mental health education in colleges and universities is to improve the mental health level of college students. Its fundamental goal is to fully tap the psychological potential of college students, cultivate their good psychological quality, promote the sound development of their personality, and enhance their social adaptability. Mental health education should not only stay on one-to-one counseling but also carry out active mental health education, so as to get good results. College students' thoughts change with their age, so it is necessary to teach students in accordance with their aptitude according to the characteristics of each grade, so as to achieve practical results. In terms of curriculum content, courses such as communicative psychology, social psychology, and positive psychology can be added. Each department should be equipped with at least one full-time mental health education teacher, set up a college students' mental health consultation association, and take the initiative to pay attention to the psychological counseling and consultation work of students with academic difficulties, students with emotional problems, graduates with employment difficulties, and students with introverted personality, so as to help them overcome psychological obstacles and reduce stress.

### 3.2. Improve the Mental Health Education System

The way of university education is classroom education, so the mental health education is also taught through the way of university classroom, which requires that the mental health education in university must be diversified, multilevel, and targeted. According to the different development stages of students, in the course of mental health education, colleges and universities should actively organize mental health educators to carry out targeted theoretical teaching. The theoretical teaching content should reflect the characteristics of higher vocational education, such as healthy professional personality education, postenvironment psychological adaptation education, interpersonal harmony education, postfrustration psychological education, and so on. In addition to daily work, psychological health education consulting institutions in colleges and universities should work hand in hand with classroom psychological health education to do a good job in psychological counseling and management for students' development, study, making friends, falling in love, and seeking jobs. The Ministry of Education should start from the source, establish a complete psychological education institution, improve the psychological health education system, and improve the professional quality of psychological educators.

Mental health education in schools is a systematic educational process, which should improve the whole process, from curriculum setting to students' psychological counseling, and improve the responsible persons and counseling procedures of each link, so that the mental health guidance work in colleges and universities can really operate.  Figure 3 shows the theoretical framework of college students' entrepreneurial team competence.

Mental health educators should take their jobs seriously and actively communicate with college students; instead of turning the psychological counseling room into a decoration, they should turn the psychological counseling room into real psychological counseling and get the recognition of students. The effect of active entrepreneurship education on college students' entrepreneurial psychological quality is shown in Figure 4.

University leaders should correct their understanding of college students' mental health education, deeply understand and carry out college students' mental health education, give support in all aspects, encourage and advocate college students to actively communicate with relevant psychological educators when they encounter problems, and boldly speak out their problems and their true inner thoughts. Colleges and universities should strive to create a strong cultural and educational atmosphere of mental health, let students actively participate in activities, and enhance the mental health awareness of the new concept of health. Schools should integrate mental health education into the overall work of schools, so as to enable students to establish positive mental health awareness and abandon conservative and backward concepts. To strengthen the standardized management of college students' mental health education, it is necessary to bring it into the educational system of colleges and universities. The specific implementation can be managed by subprincipals, set up a special working group on mental health education, and formulate working rules and regulations.

## 4. Conclusions

As a special social group, college students face many psychological problems. If they cannot be guided and solved in time, they will cause psychological problems and affect their healthy development. College students' mental health problems have certain complexity, and it is an inevitable requirement of talent cultivation in colleges and universities to carry out mental health education for college students. The way of university education is classroom education, so the mental health education is also taught through the way of university classroom, which requires that the mental health education in university must be diversified, multilevel, and targeted. In carrying out mental health education for college students, colleges and universities are actively exploring effective ways to achieve it. Of course, there are still some problems, which need to further strengthen mental health education measures for college students to promote their physical and mental health development. Colleges and universities should focus on carrying out various tasks of mental health education for college students, so as to improve the actual effect of mental health education for college students. Colleges and universities must take it seriously, improve the mechanism, create a good environment, and do a good job in mental health education for college students, so as to promote the healthy growth of college students.

## Figures and Tables

**Figure 1:** Interactive relationship between students' social development.

**Figure 2:** The evolutionary structure of college students' psychological crisis.

**Figure 3:** The theoretical framework of entrepreneurial team competence.

**Figure 4:** The effect of active entrepreneurial psychological education on the improvement of college students' entrepreneurial psychological quality.

**Table 1:** Survey of psychological training plans.

	Number of people	Proportion (%)
Make a systematic psychological training plan	52	13
Arrange according to experience	348	87

## Data Availability

The data used to support the findings of this study are included within the article.
